The article "Nitrogen and potassium application effects on productivity, profitability and nutrient use efficiency of irrigated wheat (Triticum aestivum L.)" was retracted in 2025. Reasons: unreliable results or conclusions; concerns about the article.

# Nitrogen and potassium application effects on productivity, profitability and nutrient use efficiency of irrigated wheat (*Triticum aestivum* L.)

**DOI:** 10.1371/journal.pone.0264210

**Published:** 2022-05-24

**Authors:** Sandeep Sharma, Gagandeep Kaur, Pritpal Singh, Saud Alamri, Ritesh Kumar, Manzer H. Siddiqui

**Affiliations:** 1 Department of Soil Science, Punjab Agricultural University, Ludhiana, India; 2 Yadvindra Department of Engineering, Punjabi University South Campus, Talwandi Sabo, Bathinda, Punjab, India; 3 Department of Botany and Microbiology, College of Science, King Saud University, Riyadh, Saudi Arabia; 4 Department of Agronomy, Kansas State University, 2004 Throckmorton Plant Science Center, Manhattan, KS, United States of America; COMSATS University Islamabad (CUI), PAKISTAN

## Abstract

The development of robust nutrient management strategies have played a crucial role in improving crop productivity, profitability and nutrient use efficiency. Therefore, the implementation of efficient nutrient management stratigies is important for food security and environmental safety. Amongst the essential plant nutrients, managing nitrogen (N) and potassium (K) in wheat (*Triticum aestivum* L.) based production systems is citically important to maximize profitable production with minimal negative environmental impacts. We investigated the effects of different fertilizer-N (viz. 0–240 kg N ha^-1^; N_0_-N_240_) and fertilizer-K (viz. 0–90 kg K ha^-1^; K_0_-K_90_) application rates on wheat productivity, nutrient (N and K) use efficiency viz. partial factor productivity (PFP_N/K_), agronomic efficiency (AE_N/K_), physiological efficiency (PE_N/K_), reciprocal internal use efficiency (RIUE_N/K_), and profitability in terms of benefit-cost (B-C) ratio, gross returns above fertilizer cost (GRAFC) and the returns on investment (ROI) on fertilizer application. These results revealed that wheat productivity, plant growth and yield attributes, nutrients uptake and use efficiency increased significantly (*p<*0.05)with fertilizer-N application, although the interaction effect of N x K application was statistically non-significant (*p<*0.05). Fertilizer-N application at 120 kg N ha^-1^ (N_120_) increased the number of effective tillers (8.7%), grain yield (17.3%), straw yield (15.1%), total N uptake (25.1%) and total K uptake (16.1%) than the N_80_. Fertilizer-N application significantly increased the SPAD reading by ~4.2–10.6% with fertilizer-N application (N_80_-N_240_), compared with N_0_. The PFP_N_ and PFP_K_ increased significantly with fertilizer-N and K application in wheat. The AE_N_ varied between 12.3 and 22.2 kg kg^-1^ with significantly higher value of 20.8 kg kg^-1^ in N_120_. Fertilizer-N application at higher rate (N_160_) significantly decreased the AE_N_ by ~16.3% over N_120_. The N_120_treatment increased the AE_K_ by ~52.6% than N_80_ treatment. Similarly the RIUE_N_ varied between 10.6 and 25.6 kg Mg^-1^ grain yield, and increased significantly by ~80.2% with N_120_ as compared to N_0_ treatment. The RIUE_K_ varied between 109 and 15.1 kg Mg^-1^ grain yield, and was significantly higher in N_120_ treatment. The significant increase in mean gross returns (MGRs) by ~17.3% and mean net returns (MNRs) by ~24.1% increased the B-C ratio by ~15.1% with N_120_ than the N_80_ treatment. Fertilizer-N application in N_120_ treatment increased the economic efficiency of wheat by ~24.1% and GRAFC by ~16.9%. Grain yield was significantly correlated with total N uptake (r = 0.932**, *p*<0.01), K uptake (r = 0.851**), SPAD value (r = 0.945**), green seeker reading (r = 0.956**), and the RIUE_N_ (r = 0.910**). The artificial neural networks (ANNs) showed highly satisfactory performance in training and simulation of testing data-set on wheat grain yield. The calculated mean absolute error (MAE), mean absolute percentage error (MAPE) and root mean square error (RMSE) for wheat were 0.0087, 0.834 and 0.052, respectively. The well trained ANNs model was capable of producing consistency for the training and testing correlation (R^2^ = 0.994**, *p*<0.01) between the predicted and actual values of wheat grain yield, which implies that ANN model succeeded in wheat grain yield prediction.

## 1. Introduction

Wheat (*Triticum aestivum* L.) is extensively utilized in human consumption and has high rank globally among the most essential cereals grown worldwide. It accounts for ~30% of all cereal food worldwide and staple food for ~10 billion people in ~43 countries of the world [1, 2]. The most important factors influencing the wheat grain quality parameters are the environment, genotype and the potential interactions among these factors [3, 4]. Nitrogen is most important yield limiting nutrients for crop growth in different agro-ecological regions. Fertilizer-N affect the physiological (i.e. respiration rate, water balance, signaling pathways) [5] and metabolic (i.e. enzyme activity, photosynthesis rate) processes of plants, which influencing plant growth [6, 7]. Research on N fertilization to cereal crops has been well highlighted because of its essential role in high yielding systems [8–10], improved dough quality and the potential for environmental impacts due to low N use efficiency [10, 11].

After N, potassium (K) is absorbed in large amount than any other element [12] and plays a lead role in increasing crop yield and improving the product quality [13, 14]. Potassium supply is considered as a limiting factor, given its high accumulation in cereals [15, 16]. Fertilizer-K application is required for plant survival, carbohydrate and proteins syntheses, cell evolution which helps in maintaining the ionic cell balance and acts as an enzyme activator besides activating the photosynthetic enzymes, assimilates translocation [17, 18] and enhance stress tolerance [19, 20]. Potassium effectively coordinates the relationship between source and sink of starch synthesis and transport and transformation of photosynthates [21]. But, imbalanced fertilizer application in crop production has become common in many developing countries [10, 22, 23]. The practice often leads to an excess of fertilizer-N application with a serious environmental implications [24], besides continual depletion of soil K mainly due to inadequate K supply [22]. Over application of fertilizer-N leads to enrichment of reactive N constituents, transformation of soil N forms and also affects soil acidification, with resultant impairment of ecosystems [24, 25]. Bijay-Singh et al. [26] reported that to a large percentage of area under rice-wheat system, very little or no fertilizer-K is being applied and therefore, most of it comes from K-reserves of the soil. There are many causes of low K use in farmers’ fields, such as the effect of K in vegetative crop growth is not very clear, K fertilizer are more costly than fertilizer-N, and sometimes it is not available in the local market [27].

The apparent recovery of nutrients from applied fertilizers for cereal crops is typically low [28, 29]. Recent evidence suggests that the co-application of fertilizers (P, K and S) can improve the recovery of fertilizer-N and increased N efficiency [30]. The causes of yield gaps due to nutrient deficiencies and imbalances among regions can be enhanced yields ~20–30%, by management practices [31]. Therefore, a better characterization of wheat response to fertilizer application and interactions among nutrients is essential for sustainable improvements in yield [32]. While extensive research has explored the wheat response to fertilizer-N, P, and K over the years, but with few exceptions [33, 34] most studies were usually limited in geography [35, 36] or on temporal scale [36, 37]. Fertilizer-N application intensifies K requirement of crops due to yield gain benefits, therefore, high K application rates become essential to achieve higher crop yields [38]. Contrarily, increasing fertilizer-N application to crops with insufficient soil K status could increase K recycling from the deep layers. Therefore, the fertilizer-N and K application rates must be adjusted to optimize and rationalize crop demand and reduce the negative impacts on soils’ K reserves due to high K mining [39].

While extensive research has explored wheat crop response to fertilizer-N, P, and K over the years [36, 37] but provided a limited potential to extrapolate the interactive effect of N and K on wheat yield and nutrient use efficiency. Additionally, despite potential interaction effects of fertilizer rates (N, P, and K) on crop’s responses [38], most studies focused on one nutrients at a time [30, 39], and very few studies attempted to explore the interaction effects among fertilizer-N, and K applications [33]. Wheat yield response to fertilizer-K depends on the N nutrition level and the interaction is usually positive [40]. Nonetheless, fertilizer-K application facilitates the absorption and transport of nitrate-N (NO^3—^N) to the shoots of the plant and transports it later on to the aerial plant parts, which in turn increases the activities of N [41, 42]. The availability and proper ratio in the soil are important factors for plant growth and development [38]. In addition, changes in NH_4_^+^/NO_3_^−^ ratios and K supply levels influence the yield and nutrient uptake of wheat [43]. Therefore, interaction effect of fertilizer-N and K can be assessed by with wide range of fertilizer application rates of two or more nutrients on nutrient uptake, yield and nutrient use efficiency. A better understanding of fertilizer-N and -K interactions affecting crop yield and nutrient use efficiency has important agronomic consequences in economic and environmental context. Therefore, the objective of this field experiment was to investigate fertilizer-N by K interaction in wheat by evaluating the effects of wide range of fertilizer-N and K applications in different combinations on yield, nutrient use efficiency and economic indices in irrigated sandy loam ellitic soil in north-western India.

## 2. Results

### 2.1. Yield attributes and crop productivity

Fertilizer-N application significantly (*p*<0.05) increased the number of effective tillers and non-effective tillers during 2 study years, while fertilizer-K application did not increased the number of effective tillers of wheat (Table 1). Data pooled for study years showed that N_160_ increased the number of effective tillers by ~3.4-times, compared with the N_0_. Similarly, N_160_ increased the number of non-effective tillers significantly over the N_0_. At higher fertilizer-N applications, the number of effective and non-effective tillers did not increased significantly. The plant height and spike length did not increased significantly with fertilizer-N and K application. The root dry weight increased significantly by 25.6 g plant^-1^ (~164%) with N_120_ compared with N_0_. The interaction effect of fertilizer-N and K application on yield attributes of wheat was statistically non-significant. Fertilizer-N application increased the root dry weight up to fertilizer-N application rate of 120 kg N ha^-1^, and thereafter there was no change in the root dry weight (Fig 1). The relationship between fertilizer-N application rates and root dry weight of wheat could best be expressed as Eq 1.


$$Root\;dry\;weight\;(g\;plant^{‐1})=‐0.0001\;{\left(Fertilizer‐N,\;kg\;N\;ha^{‐1}\right)}^{2}+0.302\;(Fertilizer‐N,\;kg\;N\;ha^{‐1})+16.74,\;R^{2}=0.959$$ (1)

**Fig 1:** Relationship between fertilizer-N application rate (kg N ha^-1^) and dry root weight (g plant^-1^) of wheat (*Triticum aestivum* L.) in a sandy loam soil. *Line bars indicate standard error from mean (S*.*E*._*M*_).

**Table 1:** Effect of nitrogen (N) and potassium (K) application on yield attributes viz. number of effective tillers, number of non-effective tillers, plant height, spike lengh and root drt weight of wheat (*Triticum aestivum* L.) in a sandy loam soil in sub-tropical India.

Treatment	Effective tillers (No. 2m^-1^ row length)			Non-effective tillers (No. 2m^-1^ row length)			Plant height (cm)			Spike length (cm)			Root dry weight (g plant^-1^)		
	2012	2013	Pooled	2012	2013	Pooled	2012	2013	Pooled	2012	2013	Pooled	2012	2013	Pooled
Main plot (N application)															
N_0_	55	59	57	11.7	14.2	12.9	70.7	66.8	68.2	6.9	7.1	6.9	16.5	14.4	15.6
N_80_	170	175	172	22.3	24.7	23.1	90.1	92.7	91.2	9.1	8.6	8.8	38.1	40.2	38.8
N_120_	184	193	187	22.5	25.9	24.1	107.1	104.5	105.4	9.3	8.9	9.1	39.4	42.5	41.2
N_160_	190	199	194	25.2	28.7	26.7	104.5	108.6	106.2	8.9	9.2	9.0	40.3	43.2	41.9
N_200_	203	210	207	26.3	30.2	27.9	105.5	107.6	106.2	9.0	9.4	9.2	41.2	42.9	42.1
N_240_	207	213	210	27.6	31.4	28.8	107.5	111.2	108.4	9.2	9.6	9.4	42.0	44.7	43.5
LSD (*p<*0.05)	18.4	19.1	18.7	3.7	1.8	1.9	NS	NS	NS	NS	NS	NS	3.1	3.4	3.2
Sub-plot (K application)															
K_0_	165	172	167	22.0	24.1	23.1	96.8	93.9	94.5	9.3	8.7	9.1	36.5	34.7	35.4
K_30_	171	181	175	23.0	25.7	24.6	97.6	99.5	98.3	8.2	8.7	8.5	36.1	38.4	37.3
K_60_	169	179	173	22.6	26.4	25.6	99.4	102.4	101.2	9.5	8.9	9.2	36.3	38.9	37.4
K_90_	168	179	174	22.7	26.8	26.1	100.1	103.8	102.4	8.2	8.9	8.6	36.2	38.5	37.6
LSD (*p<*0.05)	NS	NS	NS	NS	NS	NS	NS	NS	NS	NS	NS	NS	NS	NS	NS

Wheat grain yield increased significantly up to N_120_ during 2014, while in 2013 the significant increase was observed up to N_160_ (Table 2). Data pooled for two years showed that wheat grain yield was increased by 2.5 Mg ha^-1^ (~76.5%) with N_120_, compared with N_0_. Similarly, straw yield did not increased significantly with N_160_ than the N_120_. The fertilizer-N and K application did not significantly increase the harvest index of wheat. The interaction effect of fertilizer-N and K on wheat grain and the harvest index was non-significant. Fertilizer-K application at K_90_ resulted in significant increase in wheat straw yield. Fig 2 illustrates that wheat grain yield increased in non-linear way with fertilizer-N application, and the relationship between fertilizer-N application rates and wheat grain yield could best be described by Eq 2.


$$Wheat\;grain\;yield\;(Mg\;ha^{‐1})=‐6E‐05\;{\left(Fertilizer‐N,\;kg\;N\;ha^{‐1}\right)}^{2}+0.027\;(Fertilizer‐N,\;kg\;N\;ha^{‐1})+3.244,\;R^{2}=0.994$$ (2)

**Fig 2:** Relationship between fertilizer-N application rate (kg N ha^-1^)and grain yield (Mg ha^-1^) of wheat (*Triticum aestivum* L.) in a sandy loam soil. *Line bars indicate standard error from mean (S*.*E*._*M*_).

**Table 2:** Effect of nitrogen (N) and potassium (K) application on wheat grain, straw yield (Mg ha^-1^) and harvest index in a sandy loam soil in sub-tropical India.

Treatment	Grain yield (Mg ha^-1^)			Straw yield (Mg ha^-1^)			Harvest index (HI)		
	2012	2013	Pooled	2012	2013	Pooled	2012	2013	Pooled
Main plot (N application)									
N_0_	3.28	3.26	3.27	3.61	3.32	3.47	0.48	0.50	0.49
N_80_	5.05	4.79	4.92	6.57	6.15	5.74	0.43	0.44	0.46
N_120_	5.67	5.87	5.77	7.43	6.78	6.60	0.43	0.46	0.47
N_160_	5.57	6.55	6.06	7.39	6.79	6.73	0.43	0.49	0.47
N_200_	5.57	6.78	6.17	7.71	7.17	6.94	0.42	0.49	0.47
N_240_	5.44	7.00	6.22	7.61	7.54	6.92	0.42	0.48	0.47
LSD (*p*<0.05)	0.59	0.31	0.30	0.61	0.80	0.74	NS	NS	NS
Sub-plot (K application)									
K_0_	5.25	6.30	5.78	7.03	6.87	6.40	0.43	0.48	0.47
K_30_	5.44	6.10	5.77	7.28	6.72	6.53	0.43	0.48	0.47
K_60_	5.53	6.21	5.87	7.45	6.91	6.66	0.43	0.47	0.47
K_90_	5.61	6.17	5.89	7.61	7.04	6.75	0.42	0.47	0.47
LSD (*p<*0.05)	NS	NS	NS	0.34	0.35	0.34	NS	NS	NS

### 2.2. Nutrient uptake and leaf greenness

Fertilizer-N application significantly increased the grain, straw and total (grain + straw) N uptake by wheat during the study years (Table 3). Grain N uptake increased significantly with N_160_ compared with N_120_ during the second years, but non-significantly during the first year. Data pooled for two study years revealed that grain N uptake was significantly increased with N_160_ than the N_120_. Grain-N uptake was increased by ~3.5 and 4.0-times with N_120_ and N_160_, respectively over the N_0_. As compared with N_120_, N_160_ resulted in ~15.5% increase in grain N uptake by wheat. The highest straw N uptake was observed with N_240_; although N_120_ and N_160_ increased the straw N uptake by ~2.8 and 3.1-times than the N_0_. The total N uptake by wheat varied between 33.3 and 158.4 kg ha^-1^; showing an increase of ~3.8 and 4.0-times with N_120_ and N_160_ over N_0_.

**Table 3:** Effect of nitrogen (N) and potassium (K) application on N uptake by grain and straw of wheat (*Triticum aestivum* L.) in a sandy loam soil in sub-tropical India.

Treatment	Grain N uptake (kg ha^-1^)			Straw N uptake (kg ha^-1^)			Total N uptake (kg ha^-1^)		
	2012	2013	Pooled	2012	2013	Pooled	2012	2013	Pooled
Main plot (N application)									
N_0_	25.7	24.7	25.2	7.1	9.1	8.1	32.8	33.7	33.3
N_80_	71.9	64.8	68.3	19.9	19.1	19.5	91.8	83.9	87.8
N_120_	88.1	86.6	87.3	23.1	21.8	22.5	111.2	108.4	109.8
N_160_	95.1	106.4	100.8	25.9	24.1	25.0	121.0	130.5	125.7
N_200_	99.0	114.5	106.8	28.1	26.6	27.4	127.2	141.1	134.1
N_240_	110.8	135.6	123.2	35.1	35.5	35.3	145.8	171.1	158.4
LSD (*p<*0.05)	12.9	12.7	12.1	5.1	5.3	4.9	16.9	15.5	15.2
Sub-plot (K application)									
K_0_	79.7	91.4	85.5	23.1	23.3	23.2	102.8	114.7	108.7
K_30_	83.9	89.4	86.7	22.6	21.9	22.3	106.5	111.3	108.9
K_60_	83.5	89.9	86.7	22.8	22.0	22.4	106.3	112.0	109.1
K_90_	80.0	84.3	82.1	24.3	23.5	23.9	104.3	107.8	106.0
LSD (*p<*0.05)	NS	NS	NS	NS	NS	NS	NS	NS	NS

These results revealed that increased fertilizer-N rate of N_160_ resulted in only ~6.7% increase in total N uptake by wheat. It was important to note that fertilizer-K application did not result in significant change in total N uptake by wheat. The interaction effect of fertilizer-N and K application was statistically non-significant.

Fertilizer-N application significantly increased the SPAD reading by ~4.2–10.6% with fertilizer-N application (N_80_-N_240_), compared with N_0_ (Fig 3). At higher fertilizer-N rate (N_160_) the SPAD reading increased by ~2.3%, compared with N_120_. Fertilizer-K application did not significantly change the SPAD reading. The green seeker value followed the similar trend to that of the SPAD reading, with no significant change due to fertilizer-K application. Fig 4 illustrates the relationship between SPAD value and grain, straw and total N uptake by wheat. The relationship indicates increase in N uptake with the increase in SPAD value, which could best be described by Eqs 3–5.


$$Grain\;N\;uptake\;(kg\;N\;ha^{‐1})=‐2.526{\;(SPAD\;reading)}^{2}+217.0\;(SPAD\;reading)‐4540,\;R^{2}=0.971$$ (3)

$$Straw\;N\;uptake\;(kg\;N\;ha^{‐1})=‐0.36{\;(SPAD\;reading)}^{2}+32.98\;(SPAD\;reading)‐716.9,\;R^{2}=0.941$$ (4)

$$Total\;N\;uptake\;(kg\;N\;ha^{‐1})=‐2.888{\;(SPAD\;reading)}^{2}+250.1\;(SPAD\;reading)‐5259,\;R^{2}=0.969$$ (5)

**Fig 3:** Effect of nitrogen (N) and potassium (K) application on SPAD value of wheat (*Triticum aestivum* L.) in a sandy loam soil in sub-tropical India. *Bars indicate the standard error from mean (S*.*E*._*M*_*)*.

**Fig 4:** Quantitative relationship between SPAD value and N uptake (kg ha^-1^) by grain, straw and total (grain + straw) N uptake by wheat (*Triticum aestivum* L.) in a sandy loam soil.

Fig 5 showed the green seeker value in response to fertilizer-N application in wheat. The N uptake exhibited an increase as a function of green seeker reading (Fig 6). The relationship between green seeker reading and N uptake by straw, grains and total N uptake has been expressed in Eqs 6–8.


$$Grain\;N\;uptake\;(kg\;N\;ha^{‐1})=153.6{\;(green\;seeker\;reading)}^{6.377},\;R^{2}=0.890$$ (6)

$$Straw\;N\;uptake\;(kg\;N\;ha^{‐1})=0.876{\;(green\;seeker\;reading)}^{5.542},\;R^{2}=0.876$$ (7)

$$Total\;N\;uptake\;(kg\;N\;ha^{‐1})=191.7{\;(green\;seeker\;reading)}^{6.188},\;R^{2}=0.890$$ (8)

**Fig 5:** Effect of nitrogen (N) and potassium (K) application on green seeker value for wheat (*Triticum aestivum* L.) in a sandy loam soil in sub-tropical India. *Bars indicate the standard error from mean (S*.*E*._*M*_*)*.

**Fig 6:** Quantitative relationship between Green seeker value and N uptake by grain, straw and total (grain + straw) N uptake by wheat (*Triticum aestivum* L.) in a sandy loam soil.

Fertilizer-N application resulted in a significant increase in K uptake by grains and straw (Table 4). Data pooled for two years showed that grain K uptake varied between 11.8 and 22.3 kg ha^-1^; with ~84.7% increase in N_120_ than the N_0_ treatment. There was non-significant difference in grain K uptake at higher fertilizer-N rates (N_160_-N_240_). These results showed that wheat straw K uptake was significantly increased with N_120_; followed by non-significant change at higher fertilizer-N rates. The total K uptake followed the similar response to fertilizer-N application, with highest K uptake at N_120_. Data pooled for different study shows that there was non-significant difference in grain, straw and total K uptake with different rates of fertilizer-K application. Nonetheless, the interaction effect of fertilizer-N and K on K uptake by grains and straw was non-significant.

**Table 4:** Effect of nitrogen (N) and potassium (K) application on K uptake by grain and straw of wheat (*Triticum aestivum* L.) in a sandy loam soil in sub-tropical India.

Treatment	Grain K uptake (kg ha^-1^)			Straw K uptake (kg ha^-1^)			Total K uptake (kg ha^-1^)		
	2012	2013	Pooled	2012	2013	Pooled	2012	2013	Pooled
Main plot (N application)									
N_0_	11.9	11.7	11.8	23.2	24.5	23.9	35.1	36.3	35.7
N_80_	21.5	21.0	21.3	52.7	51.6	52.2	74.2	72.6	73.4
N_120_	21.1	22.5	21.8	61.8	65.0	63.4	82.9	87.5	85.2
N_160_	19.9	24.0	21.9	59.3	57.3	58.3	79.2	81.3	80.3
N_200_	19.7	24.8	22.2	62.8	61.5	62.1	82.5	86.3	84.4
N_240_	19.2	25.5	22.3	69.0	72.0	70.5	88.2	97.5	92.8
LSD (*p<*0.05)	3.3	2.93	2.9	11.8	11.9	10.7	12.3	13.3	11.3
Sub-plot (K application)									
K_0_	17.7	21.4	19.5	52.3	58.1	55.2	70.0	79.5	74.7
K_30_	19.3	21.9	20.6	50.6	49.3	50.0	70.0	71.2	70.6
K_60_	19.0	21.5	20.3	57.2	56.6	56.9	76.3	78.1	77.2
K_90_	19.5	21.6	20.5	59.1	57.3	58.2	78.5	78.9	78.7
LSD (*p<*0.05)	1.6	NS	NS	NS	9.5	NS	NS	NS	NS

### 2.3. Nitrogen and potassium use efficiency

The PFP_N_ decreased significantly with increased fertilizer-N application rate in wheat, but do not differ significantly with the application of fertilizer-K (Table 5). Data pooled for different study years showed that PFP_N_ for wheat varied between 25.9 and 61.5 kg ha^-1^; with the highest in N_80_ and the lowest in N_240_. The N_160_ treatment decreased the PFP_N_ by 10.1 kg ha^-1^ (~21.0%), compared with N_120_. The AE_N_ varied between 12.3 and 22.2 kg kg^-1^ with significantly higher value of 20.8 kg kg^-1^ in N_120_. Fertilizer-N application at higher rate (N_160_) significantly decreased the AE_N_ by ~16.3% over N_120_. The two year pooled data showed that PE_N_ was significantly higher with N_120_ by ~44.6% than the N_240_. It was important to observe that PE_N_ did not differ significantly among N_120_ and N_160_. The RIUE_N_ varied between 10.6 and 25.6 kg Mg^-1^ grain yield, and increased significantly by ~80.2% with N_120_ as compared to N_0_ treatment. The RIUE_N_ did not differ significantly among N_120_ and N_160_. The effect of fertilizer-K and interaction effect of fertilizer-N and K was statistically non-significant for PFP_N_, AE_N_, PE_N_ and the RIUE_N_.

**Table 5:** Effect of nitrogen (N) and potassium (K) application on N use efficiency in wheat (*Triticum aestivum* L.) in a sandy loam soil in sub-tropical India.

Treatment	Partial factor productivity (PFP_N_; kg ha^-1^)			Agronomic efficiency (AE_N_; kg kg^-1^)			Physiological efficiency (PE_N_; kg kg^-1^)			Reciprocal interval use efficiency (RIUE_N_; kg Mg^-1^ grain yield)		
	2012	2013	Pooled	2012	2013	Pooled	2012	2013	Pooled	2012	2013	Pooled
Main plot (N application)												
N_0_	--	--	--	--	--	--	--	--	--	10.0	11.1	10.6
N_80_	63.1	59.9	61.5	22.1	22.4	22.2	30.4	34.3	32.3	18.2	17.5	17.9
N_120_	47.2	48.9	48.0	19.9	21.7	20.8	30.9	37.2	34.1	19.6	18.5	19.1
N_160_	34.8	41.0	37.9	14.3	20.6	17.4	26.0	35.8	30.9	21.8	19.9	20.9
N_200_	27.8	33.9	30.9	11.4	17.6	14.5	24.6	34.7	29.6	22.8	20.9	21.9
N_240_	22.7	29.2	25.9	9.0	15.6	12.3	19.3	28.0	23.6	26.8	24.4	25.6
LSD (*p<*0.05)	6.2	2.1	3.5	5.1	2.1	2.9	3.5	3.2	3.4	1.2	2.4	2.2
Sub-plot (K application)												
K_0_	37.6	43.2	40.4	12.1	18.6	15.3	20.9	27.1	24.0	20.2	18.8	19.5
K_30_	39.0	41.9	40.4	12.8	15.8	14.3	21.8	27.4	24.6	20.2	18.9	19.6
K_60_	39.6	42.7	41.2	13.0	15.9	14.5	21.6	30.5	26.0	19.8	19.0	19.4
K_90_	40.2	42.5	41.4	13.1	15.0	14.1	23.2	28.3	25.8	19.3	18.1	18.7
LSD (*p<*0.05)	NS	NS	NS	NS	NS	NS	NS	NS	NS	NS	NS	NS

The PFP_K_ increased significantly with fertilizer-N and K application in wheat (Table 6). Fertilizer-N application at 120 kg N ha^-1^ increased the PFP_K_ by 38.3 kg ha^-1^ (~76.9%), compared with the N_0_ treatment. However, the PFP_K_ did not differ significantly among different fertilizer-N application rates (N_80_-N_240_). The PFP_K_ was highest at K_30_ and decreased by ~2-times with K_60_ treatment. Fertilizer-N application at N_120_ increased the AE_K_ by ~52.6% than N_80_ treatment. Similarly, K_30_ treatment had the highest, while the K_90_ had the significantly lower AE_K_. The PE_K_ was highest in N_160_, which was ~19.8% higher than N_120_ treatment. The PE_K_ did not differ significantly with fertilizer-K application at different rates. The RIUE_K_ varied between 109 and 15.1 kg Mg^-1^ grain yield, and was significantly higher in N_120_ treatment. The effect of fertilizer-K and interaction effect of fertilizer-N and K on RIUE_K_ of wheat crop statistically non-significant.

**Table 6:** Effect of nitrogen (N) and potassium (K) application on K use efficiency in wheat (*Triticum aestivum* L.) in a sandy loam soil in sub-tropical India.

Treatment	Partial factor productivity (PFP_K_; kg ha^-1^)			Agronomic efficiency (AE_K_; kg kg^-1^)			Physiological efficiency (PE_K_; kg kg^-1^)			Reciprocal interval use efficiency (RIUE_K_; kg Mg^-1^ grain yield)		
	2012	2013	Pooled	2012	2013	Pooled	2012	2013	Pooled	2012	2013	Pooled
Main plot (N application)												
N_0_	50.3	49.4	49.8	--	--	--	--	--	--	10.6	11.1	10.9
N_80_	77.3	72.6	75.0	27.1	23.2	25.1	46.2	43.2	44.7	14.6	15.1	14.9
N_120_	87.7	88.4	88.1	37.4	39.1	38.3	51.5	58.7	55.1	15.6	14.8	15.2
N_160_	86.1	100.9	93.5	35.8	51.5	43.7	56.6	75.8	66.2	14.2	12.4	13.3
N_200_	85.4	102.0	93.7	35.1	52.7	43.9	51.3	75.8	63.5	14.8	12.8	13.8
N_240_	83.1	105.6	94.3	32.9	56.2	44.5	43.3	66.2	54.7	16.2	13.9	15.1
LSD (*p<*0.05)	31.7	44.1	34.2	NS	5.4	4.8	NS	17.7	9.3	2.1	1.7	1.8
Sub-plot (K application)												
K_0_	--	--	--	--	--	--	41.0	45.9	50.9	14.6	13.5	14.0
K_30_	169.0	187.2	178.1	60.6	81.5	71.0	39.1	45.4	51.8	13.6	12.6	13.1
K_60_	86.0	95.3	90.7	30.9	41.2	36.0	45.8	53.1	60.5	14.6	13.8	14.2
K_90_	58.2	63.4	60.8	20.7	25.8	23.3	40.1	45.0	49.9	14.6	13.6	14.1
LSD (*p<*0.05)	29.5	38.1	40.2	5.9	5.2	5.6	NS	NS	NS	NS	NS	NS

### 2.4. Available nitrogen and potassium content

Fig 7 showed that available-N content in soil was significantly increased with fertilizer-N application. The available-N content in soil increased by ~37.3% with N_120_ treatment compared with the N_0_. There was non-significant change in available-N content in soil with fertilizer-N application rates of N_120_, N_160_, N_200_ and N_240_. Fertilizer-K application had non-significant effect on available-N content in soil. Available-K content in soil was highest in N_120_treatment, and was ~8.3% higher than N_0_ (Fig 8). Fertilizer-K application at K_30_, K_60_ and K_90_ increased the available-K content in soil by ~9.1, 11.5 and 15.3%, respectively.

**Fig 7:** Effect of nitrogen (N) and potassium (K) application on available-N content in a sandy loam soil in sub-tropical India. *Bars indicate the standard error from mean (S*.*E*._*M*_*)*.

**Fig 8:** Effect of nitrogen (N) and potassium (K) application on available-K content in a sandy loam soil in sub-tropical India. *Bars indicate the standard error from mean (S*.*E*._*M*_*)*.

### 2.5. Economic analysis

The MCCIs varied between 364 US$ ha^-1^ and 408 US$ ha^-1^ yielded MGRs of 835 US$ ha^-1^ and 1594 US$ ha^-1^ for different fertilizer-N and K application treatments in wheat (Table 7). The MGRs were significantly higher by ~17.3% with N_120_ as compared to N_80_. The application of higher fertilizer-N application rates did not significantly increased the MGRs for wheat cultivation. The MNRs varied between 471 US$ ha^-1^ for N_0_ and 1187 US$ ha^-1^ for N_240_ treatments. Similarly, the MNRs varied between 1115 and 1130 US$ ha^-1^ among different fertilizer-K treatments (K_0_-K_90_). Fertilizer-N application at 120 kg N ha^-1^ (N_120_) resulted in significantly higher MNRs by ~24.1% than the N_80_ treatment. The B-C ratio was significantly increased by ~66.1% with N_120_ than the N_0_ treatment. The higher fertilizer-N application rates (N_160_-N_240_) resulted in ~1.4–3.4% increase in B-C ratio of wheat. The economic efficiency of wheat increase by ~24.1% with N_120_ than N_80_ treatments; however, the higher fertilizer-N application rates did not significantly increase the economic efficiency. The GRAFC varied between 835 and 1550 US$ ha^-1^; a significantly higher returns (by ~210 US$ ha^-1^; ~16.9%) were obtained under N_120_ than N_80_. The ROI of 66.9 US$ gross returns US$^-1^ cost were significantly higher by ~84.8% in N_120_ than the N_240_ treatment. At lower fertilizer-N application rate (N_80_), the ROI although increased by ~23.3%, but were statistically non-significant.

**Table 7:** Effect of nitrogen (N) and potassium (K) application on economic indices viz. mean cost of cash inputs (MCCIs), mean gross returns (MGRs), mean net returns (MNRs), benefit-cost (B-C) ratio, economic efficiency, gross returns above the fertilizer cost (GRAFC) and returns on investment on fertilizer application (ROI) for wheat (*Triticum aestivum* L.) cultivation in a sandy loam soil in sub-tropical India. (*Data pooled for two study years*).

Treatment	MCCIs (US$ ha^-1^)	MGRs (US$ ha^-1^)	MNRs (US$ ha^-1^)	B-C ratio	Economic efficiency (US$ ha^-1^ d^-1^)	GRAFC (US$ ha^-1^)	ROI (US$ gross returns US$^-1^ cost)
Main plot (N application)							
N_0_	364	835	471	2.30	3.08	835	--
N_80_	378	1256	877	3.32	5.73	1241	85.5
N_120_	386	1473	1088	3.82	7.11	1451	66.9
N_160_	393	1551	1158	3.95	7.57	1522	52.8
N_200_	400	1580	1180	3.95	7.71	1544	43.0
N_240_	408	1594	1187	3.91	7.76	1550	36.2
LSD (*p<*0.05)		125.9	103.4	0.32	1.8	105.4	19.1
Sub-plot (K application)							
K_0_	364	1479	1115	4.07	7.29	1479	--
K_30_	368	1476	1108	4.01	7.24	1471	337.6
K_60_	372	1502	1130	4.04	7.39	1494	171.8
K_90_	377	1507	1130	4.00	7.39	1494	114.9
LSD (*p<*0.05)		NS	NS	NS	NS	NS	65.4

### 2.6. Relationship between potassium fractions, crop yields and potassium uptake

Correlation matrix revealed that wheat grain yield was highly correlated with grain N uptake (r = 0.924**, *p*<0.01), straw N uptake (r = 0.831**, *p*<0.01), grain K uptake (r = 0.825**, *p*<0.01), straw K uptake (r = 0.838**, *p*<0.01), total N uptake value (r = 0.932**, *p*<0.01) and total K uptake (r = 0.851**, *p*<0.01) (Fig 9). Wheat grain yield also exhibited a significant linear relationship with SPAD value (r = 0.945**, *p*<0.01), green seeker reading (r = 0.956**, *p*<0.01), RIUE_N_ (r = 0.910**, *p*<0.01). We tested different regression models (Table 8) to improve the prediction of wheat grain yield by including several yield attributes. A regression model included grain and straw N and K uptake, RIUE_N_ and RIUE_K,_ SPAD and green seeker values explained ~85.3–98.4% of the wheat grain yields.

**Fig 9:** Correlation matrix depicting relationships between different variables and wheat grain yield (r > 0.435; significant at *p*<0.05 and r > 0.802 significant at *p*<0.01, others non-significant).

**Table 8:** Stepwise regression among different variables for predicting wheat (*Triticum aestivum* L.) grain yield.

Response	Regression equation	R^2^_*adj*_	R^2^	F value	*p* (<0.05)
Y_1_	2.698+0.031X_1_	0.847	0.853	127.9	0.0001^a^
Y_2_	2.511+0.023 X_1_+0.041 X_2_	0.887	0.897	91.2	0.0002^b^
Y_3_	2.545+0.024 X_1_+0.042X_2_-0.004 X_3_	0.881	0.897	58.0	0.0001^c^
Y_4_	2.273–0.019X_1_+0.033 X_2_-0.003 X_3_+0.018 X_4_	0.905	0.921	55.5	0.0001^d^
Y_5_	2.191+0.028X_1_+0.046X_2_-0.004X_3_+0.019X_4_-0.009 X_5_	0.902	0.924	43.5	0.0002^e^
Y_6_	2.145–0.017X_1_-0.009X_2_+0.0110X_3_+0.08X_4_+0.033X_5_-0.0075X_6_	0.923	0.943	46.9	0.0001^f^
Y_7_	-3.781–0.09X_1_-0.026X_2_+0.099X_3_+0.066X_4_+0.020X_5_-0.058 X_6_+0.184X_7_	0.942	0.963	54.2	0.0001^g^
Y_8_	-9.373–0.011X_1_-0.026X_2_+0.127X_3_+0.067X_4_+0.013X_5_-0.059 X_6_+0.077X_7_+11.7X_8_	0.975	0.984	114.1	0.0001^h^
Y_9_	-9.131–0.009X_1_-0.116X_2_+0.063X_3_+0.014X_4_-0.053X_5_+0.091 X_6_+11.2X_7_-0.389X_9_	0.974	0.984	98.7	0.0001^i^

Y_1_-Y_9_ = Wheat grain yield, X_1_ = Grain N uptake, X_2_ = Straw N uptake, X_3_ = Grain K uptake, X_4_ = Straw K uptake, X_5_ = Total N uptake, X_6_ = Total K uptake, X_7_ = SPAD value, X_8_ = Green seeker value, X_9_ = RIUE_N_

### 2.7. Evaluation of ANN developed for predicting wheat grain yield

A back propagation neural network with Levenberg Marquardt algorithm was used to establish the relationship between the input variables viz. grain N uptake, straw N uptake, grain K uptake, straw K uptake, total N uptake, total K uptake, SPAD value, green seeker value, RIUE_N_ and RIUE_K_ and the wheat grain yield. We applied back propagation neural networks technique, self-organizing map (SOM) neighbour weight distance and ANNs consisted of several layers of neurons which are inter-connected and then the weights were assigned to those inter-connections (Fig 9). The SOM is an unsupervised machine learning use to produce a low-dimensional representation of a higher dimensional data-set while preserving the topological structure of the data. The SOM depicts the input data as a table with a row for each value of input variable, and columns for each variable containing each value. The SOM algorithm arranged these variables in a two-dimensional grid placing with similar variable closer together. The schematic representation of weights (weight-1 and weight-2) assigned to the inter-connections for inputs used for the simulation of wheat grain yield has been shown in Fig 10. The ANNs exhibit a highly satisfactory performance in training and simulation of testing data-set, which indicates that a well-trained ANN model is well capable of producing consistent and accurate results. This consistency between the training and testing has been clearly illustrated in Fig 11. A high correlation (R^2^ = 0.994**, *p*<0.01) between the predicted and actual values of wheat grain yield, which implies that ANN model succeeded in wheat grain yield prediction. Table 9 shows test statistics for ANN model evaluation (Fig 12). The calculated MAE, MAPE and RMSE for wheat were 0.0087, 0.834 and 0.052, respectively. The lowest possible RMSE value is zero, indicating that there is no difference between the actual and predicted data.

**Fig 10:** Schematic representation of propagation neural networks technique, self organizing map (SOM) neighbour weight distance and artificial neural networks (ANNs) consisted of several layers of neurons which are inter-connected and then the weights (weight-1 and weight-2) assigned to those inter-connections.

**Fig 11:** Schematic representation of weights (weight-1 and weight-2) assigned to the inter-connections for inputs used for the simulation of wheat grain yield using ten different input layers viz. grain N uptake, straw N uptake, grain K uptake, straw K uptake, total N uptake, total K uptake, SPAD value, green seeker value, RIUE_N_ and RIUE_K_.

**Fig 12:** Cross-correlation using scatter plot (1:1 correspondence, X = Y) of predicted and actual wheat grain (Mg ha^-1^) using Levenberg Marquardt (LM) algorithm in artificial neural networks (ANNs).

**Table 9:** Statistical criteria for evaluating the performance of artificial neural networks (ANNs) for predicting wheat grain yield under different treatments based on grain and straw N uptake, grain and straw K uptake, total N and total K uptake, SPAD value, green seeker value, and reciprocal internal use efficiency of N (RIUE_N_) and K (RIUE_K_).

Statistical index	RR^2^^†^	MAE^‡^	MAPE^¶^	RMSE^#^
Value	00.994**	00.0087	00.834	00.052

^†^R^2^ = Coefficient of determination

^‡^MAE = Mean absolute error

^¶^MAPE = Mean absolute percentage error

^#^RMSE = Root mean square error

^Δ^MBE = Mean bias error

**Significant at *p*<0.01

## 3. Discussion

The fertilizer-N application significantly (*p<*0.05) increased the number of effective and non-effective tillers during 2 study years, while fertilizer-K application did not increased the yield attributing characters of wheat. The total number of tillers increased as a function of N application rates across all levels of K rate, but peaked up at 120 kg N ha^-1^. This could be major contribution of N towards cell division, elongation and enhancing the vegetative growth, and K contribute in promoting vigorous plant growth through efficient photosynthesis [44]. The individual application effect of fertilizer-N and K on number of tillers of wheat have been reported earlier [45, 46]. Furthermore, Bundy and Andraski [47] reported the combined application of fertilizer-N and K on increased tiller production. The number of effective tillers facilitates the identification of the number of spikes that plant generates, as they can survive and produce grains [48]. The requirement for high wheat yields was influenced by population growth and development, mainly in terms of the increased tiller number per unit area [49]. The application of fertilizer-K was observed to regulate the N metabolism, which increases its absorption by the plant [50]. Therefore, when fertilizer-N and K are applied together, they enhance vegetative growth and resulted in increased number of fertile tillers per unit area.

Fertilizer-N fluxes in agro-ecosystems are important for assessing the effectiveness for wheat yield and in determining probable environmental contamination [51, 52]. The optimal fertilizer-N plays a positive role in the crop growth and productivity and helps improve the profitability and nutrient use efficiency. Some studies have shown that fertilizer-N application could increase crop yield, whereas excessive fertilizer-N aplication lead to yield reduction. In the present study, wheat grain yield increased significantly up to N_120_, compared with higher level of fertilizer-N application rates, while K application did not significantly increase the wheat grain yield. In case of control, the growth and development of plants were hampered due to imbalance uptake of essential elements, which resulted in poor performance of yield attributes and ultimately gave the lowest wheat grain yield. These findings suggested that when the rate of fertilizer-N application increased to a certain extent (N_160_-N_240_), the wheat yield would not significantly increase, but there was no-significant decline. Therefore, similar to previous research [53], these results also shows that higher fertilizer-N application rates ensured higher crop yield, but was not necessary to achieve significant yield gain advantage. Similar to the grain yield, fertilizer-N application rate significantly increased crop N accumulation compared with the N_0_ control. However, the amount of N absorbed by crops on crop yield is affected by genetic and environmental factors, compromising the relationship between fertilizer-N application rate and its accumulation in the crop [54]. Unfortunately, most farmers applied the amount of fertilizer-N based on their experience, rather than testing soil nutrients and plant growth [55]. This strongly suggests that fertilizer-N rate above 120 kg N ha^-1^, the N utilization by plants were nearly negligible and exposed to leaching, volatilization and immobilization losses. These results illustrates that combination of 120 kg N ha^-1^ with 30 kg K ha^-1^ increased the ability of plants for capturing resources and increased dry matter accumulation. In the present study, the effect of higher dose of fertilizer–K application (K_60-90_) or the interaction effect of fertilizer-N and K was statistically non-significant (*p<*0.05). The soils of studied region in north-western India are mostly containing smectite and illitic clay minerals [56]. When K is removed by plant roots from the soil solution, more K is released from the clay minerals by cation exchange. Nonetheless, average amount of K contributed to wheat through irrigation with underground water varied from 8 kg in piedmont plain to 28 kg ha^-l^ each in alluvial plain with occasional sand dune and alluvial plain with sand dune, respectively [57].

### 3.1. Nutrient uptake and leaf greenness

Fertilizer-N application significantly increased the grain, straw and total N uptake by wheat during the study years up to 120 kg N ha^-1^ as compared to higher rates of fertilizer-N application. Different rates of fertilizer-K application was showed non-significant difference in grain, straw and total K uptake. When the fertilizer-N application rate exceeds crop demand, the quantity of applied fertilizer-N used by the crops is reduced, and a larger amount of applied N remains in the soil or is lost [58]. In contrast, when the fertilizer-N rate is less than crop demand, soil N is depleted [59]. Therefore, the accumulation and loss of NO_3_^—^N in soil could be reduced by applying less amounts of fertilizer-N than or equal to that required for the optimal crop yield [25, 60].

The chlorophyll fluorescence parameters were used to estimate the function of photosynthetic apparatus and carbon assimilation rate due to its sensitivity, accessibility and non-intrusive features [61, 62]. The leaf N content has been linked directly to the chlorophyll index [63], and varied with each phenological stage [64]. The reduction in light intensity and alterations in light spectrum under fertilizer-N application rates has shown to alter chloroplast ultra-structure and chlorophyll contents [61, 65]. In this study, fertilizer-N application significantly increased the SPAD value and green seeker reading by ~4.2–10.6% and 0.89–0.97%, respectively with fertilizer-N application (N_80_-N_240_), compared with N_0_. Viana and Kiehl [38] reported that the chlorophyll index increased with fertilizer-N and potassium application. Teixeira Filho et al. [66] assessed the chlorophyll concentration in wheat plants and also reported that the fertilizer-N application rates influenced the leaf chlorophyll index, with maximum valued achieved was 46 N corresponding to the applied N dose of 147 kg N ha^-1^.

### 3.2. Nitrogen and potassium use efficiency

Nitrogen use efficiency is represented with N recovered efficiency in the crops and has a significant impact on air and water quality, biodiversity, and human health [67, 68]. The higher nutrient use efficiency is generally reflected to be the adaptation of crops to a habitat with low soil N supply [69]. In the present study, fertilizer-N application at higher rate (N_160_-N_240_) significantly decreased the N use efficiencies over N_120._ However, the K use efficiency did not differ significantly among different fertilizer-K application rates. These results corroborate earlier research findings of highest N use efficiency at the lower rate because of less losses [70, 71]. At the lower rate of fertilizer-N, the wheat plant mostly utilized the supplied N for grain yield. Hagos et al. [72] and Mesele [73] reported that that K use efficiency decreased when the rate of fertilizer-K application increases. The higher nutrient use efficiency was recorded at lower rates of fertilizer-N and K application in the present study. As reported by Bijay-Singh [74], if a unit of fertilizer to pay for its cost does not increase the yield, its use will not be economical. In addition, similar to the conclusion of Li et al. [75], the high fertilizer-N application rate (210 kg N ha^-1^) substantially decreased the N use efficiency compared to that at lower fertilizer-N application rate (52.5 kg N ha^-1^). Therefore, fertilizer-N use efficiency should be improved by farmers’ to decrease the use of high fertilizer-N rate application. Generally, NO_3_^—^N is the major source of soil N absorbed by crops [76] and the improvement of N recovery depend on the capture of by roots deep in the soil profile during the growing season [77]. Therefore, further research is looked-for to elucidate whether increasing N use efficiency through increasing utilization of residual soil NO_3_^—^N [78]. In our study, decreasing wheat yield and N use efficiency at higher fertilizer-N application rates can result in large increase in tillering and biomass production [79] and decrease the vegetative growth of organs [80], increasing lodging [81], and parasite susceptibility [82]. Numerous researchers suggested that a balanced application of fertilization can improve nutrient use efficiency and reduce environmental impacts [10, 83, 84], and that the application of fertilizers (N, P and K) results in higher grain yields [30, 85, 86]. The interaction between K and N, especially available-N and K forms on plant growth and development, has become a focus of research. Our study showed that available-N forms affect plant growth and its uptake; however, the K rate has indirectly influence on the regulation of photosynthesis and nutrient absorption, with a positive N and K interaction effects. All the N use efficiency parameters declined with increase in N rate beyond N_120_, suggesting the ideal management for higher wheat yield in this region. The increased plant dry weight and chlorophyll content is positively correlated with photosynthesis and plant growth [87]. It has been reported that application of fertilizer N in amounts more than that required to produce economic yields will lead to high N losses and low N use efficiencies [88]. The low N use efficiencies in our study suggest significant N losses or immobilization. The top dressing of fertilizer application probably resulted in much of the urea N being located on or near the soil surface, with high potential for leaching and volatilization losses of N in this slightly alkaline coarse-textured soil.

Increasing synchronization between N needed by the crop and fertilizer N supply is crucial for improving N use efficiency. Applying N when demand by the crop is high will not only increase yield but also N use efficiency [89]. Ali et al. [90] reported that fertilizer N recovery efficiency in wheat in some parts of Egypt was in the range of 35.6–51.1% by following the standard recommendation. Worldwide N recovery efficiency in cereal is reported to be ~35% [2]. Improved AE and RE of applied N support the observations of Dobermann et al. [91] who regarded AE exceeding 25 kg grain per kg applied N and RE exceeding 60% with high grain yields as efficient N management strategies for timely sown wheat. Bijay-Singh et al. [92] reported wheat response to need based fertilizer N application at MT stage. The aaccurate yield prediction requires fundamental understanding of the functional relationship between yield and these interactive factors, and to reveal such relationship requires both comprehensive datasets and powerful Algorithms [93]. The crop models and decision tools have become a crucial element of precision agriculture in the world as a result of rapid development of advanced technologies [94]. Linear regression techniques, nonlinear simulations, expert systems, Adaptive Neuro fuzzy Interference System (ANFIS), Support Vector Machines (SVM), Data Mining (DM), Genetic Programming (GP), and Artificial Neural Network (ANN) are some of the prediction methods which are used in harvest predictions under the climate change [95–97]. Among these, ANNs have been applied to model complex non-linear relations [98], and have demonstrated the capability to handle a large number of inputs and generalize correlations [99]. The ANNs have been widely used for crop yield prediction with high range of accuracy [34, 98, 100, 101]. Crop yield forecasting plays an important role in farming planning and management, domestic food supply, international food trade, ecosystem sustainability, and so on [100, 102, 103]. Amaratunga et al. [98] used Levenberg–Marquardt, Bayesian Regularization, and Scaled Conjugated Gradient algorithms to train the developed ANN model for rice grain yield prediction in Sri Lanka. They reported that Levenberg–Marquardt training algorithm has outperformed the other two algorithms in determining the relationships between climatic factors and rice grain yield with less computational time. The results were stable and satisfactory under the highly unpredicted climate scenarios. ANN relationships developed can be used to predict the future rice grain yields based on climate data from various climate models. Khosla et al. [104] applied modular ANNs for predicting the amount of monsoonal rainfall and the crop yield potential of major *kharif* crops and reported that these machine learning approach has out-perform simulation abilities. Shastry et al. [101] compared ANNs and multiple linear regression (MLR) technique for predicting wheat grain yield based on amount of rainfall, crop biomass, soil evaporation, transpiration, soil moisture, and the amount of fertilizer-N applied to the crop. The customized ANN developed by varying the number of hidden layers and number of neurons in the hidden layer and the leaning rate had shown better performance for the prediction of wheat grain yield. Guo and Xue [34] reported high inaccuracy of the spatial neural network model in wheat yield forecasting which is limited to the forecasting of crop yield only within normal ranges. They reported that caution should be taken to use neural networks when using either Nonlinear Auto-regressive Neural Network (NARNN) and Nonlinear Autoregressive with External Input Neural Network (NARXNN) model for crop yield forecasting due to their inconsistency between the results of training and forecasting. Khaki and Wang [93] reported that deep neural network (DNN) approach had advantage of state-of-the-art modeling and solution techniques with superior prediction accuracy, with a RMSE being 12% of the average yield and 50% of the standard deviation for the validation data-set using predicted weather data. With perfect weather data, the RMSE would be reduced to 11% of the average yield and 46% of the standard deviation.

## 4. Materials and methods

### 4.1. Brief description of experimental site

A 2-year field experiment (2013–14 and 2014–15) on irrigated wheat was established in 2013 starting on a *Typic Ustochrept* sandy loam soil at the experimental farm of the Punjab Agricultural University, Ludhiana, Punjab (30°56′N and 75°52′E) in the Indo Gangetic Plains (IGPs) in the north-western region of India. The surface soil (0–15 cm) layer was non-saline (electrical conductivity E.C._1:2_ = 0.24 dS m^-1^) with pH_1:2_ = 7.40 (1:2 soil: water), Walkley and Black-C = 3.46 g kg^-1^, available-N = 52.9 kg ha^-1^; 0.5 M NaHCO_3_-extractable P = 17.9 mg kg^-1^ and 1 N NH_4_OAc-extractable K = 139.8 mg kg^-1^. The study region has a sub-tropical climate, with hot, wet summers and cold dry winters. Annual mean rainfall is ~760 mm, ~80% of which received in *monsoon* season extending between July and September. Mean minimum and maximum temperatures (averaged across 30 years) during wheat (November to April) are 6.7°C and 22.6°C and in rice (June to October) are 18°C and 35°C, respectively.

### 4.2. Experimental design and treatments

The experiment was laid out in a split plot design with three replications and consisted of six fertilizer-N application rates in main-plots and four rates of fertilizer-K rates in sub-plots. The main-plot treatments consisted of six fertilizer-N application rates of 0, 80, 120, 160, 200 and 240 kg N ha^-1^ (N_0_-N_240_), and sub-plots treatments consisted of four fertilizer-K application rates of 0, 30, 60 and 90 kg Kha^-1^(K_0_-K_90_). These treatments were assigned to the same experimental plots in all the years of the study.

### 4.3. Fertilizer and irrigation management

Wheat crop received a different fertilizer-N (0, 80, 120,160, 200 and 240 kg N ha^-1^) and K (0, 30, 60 and 90 kg Kha^-1^) rates as urea (46% N) and muriate of potash (60% K_2_O). One-third of total fertilizer-N, and whole amount of fertilizer-P and fertilizer-K were drilled at wheat sowing each year. The remaining ~2/3^rd^ of fertilizer-N (as per treatment) was applied in two equal split doses immediately before first irrigation at 3 weeks and second irrigation applied at 8 weeks after sowing. Wheat was irrigated (~75 mm each) at crown root initiation, maximum tillering, panicle initiation and dough stages as recommended for the crop in the region.

### 4.4. Soil and plant analysis and estimation of nutrients use efficiencies

Soil samples from the surface (0–15 cm) soil layer were collected after the completion of two years study period. Soil samples were dried in shade and were ground and sieved through 2 mm stainless steel sieve, and stored in plastic bottles until analysis. Soil samples were analyzed for available-N and K. The grain and straw samples collected at maturity were oven-dried at 65°C for 48 h to a constant weight and ground to pass through a 0.5 mm screen. The total N and K contents were determined by micro-kjeldahl method and using flame photometry methods, respectively.

The partial factor productivity of K (PFP_N_/PFP_K_), agronomic efficiency of N and K (AE_N_/AE_N_), physiological efficiency of N and K (PE_N_/PE_K_) and the reciprocal internal use efficiency of N (RIUE_N_/RIUE_K_) were estimated using Eqs 9–16. The PFP was calculated as a ratio of grain yield (kg ha^-1^) and the total amount of fertilizer added (kg ha^-1^) using Eqs 9, 10. The AE was calculated a ratio of difference in grain yield (kg ha^-1^) in fertilizer-N and K added plots and the control (no-N/no-K) to the amount of fertilizer-N/fertilizer-K added (kg ha^-1^) using Eqs 11, 12. The PE was calculated as the ratio of difference in grain yield (total above-ground dry matter, kg ha^-1^) of fertilizer N/fertilizer-K applied and the control (no-N/no-K) to that of difference in total (grain + straw) N and K uptake (kg ha^-1^) from fertilizer applied and the control (Eqs 13, 14). The RIUE_N_ of applied N and K was calculated as the ratio of N and K uptake (kg ha^-1^) by grain to the biological yield (total above-ground dry matter, Mg ha^-1^) (Eqs 15, 16).


$${\mathrm{PFP}}_{N}({\mathrm{kg}\;\mathrm{grain}\;\mathrm{kg}}^{-1}\;\mathrm{applied})=\frac{\mathrm{Grain}\;\mathrm{yield}\;({\mathrm{kg}\;\mathrm{ha}}^{-1})}{\mathrm{Total}\;\mathrm{applied}\;({\mathrm{kg}\;\mathrm{ha}}^{-1})}$$ (9)

$${\mathrm{AE}}_{N/K}(\mathrm{kg}\;\mathrm{grains}/\mathrm{kg}\;N\;\mathrm{applied})=\frac{\left(\mathrm{Grain}\;\mathrm{yield}\;\mathrm{in}\frac{N}{K}\mathrm{fertilized}\;\mathrm{plots}\right)}{\left(\mathrm{Amount}\;\mathrm{of}\frac{N}{K}\mathrm{fertilizer}\;\mathrm{applied}\right)}$$ (10)

$${PE}_{N}/K(kg\frac{grains}{kg}N/K\;uptake)=\frac{\left(Grain\;yield\;in\;N/K\;fertilized\;plots\right)}{\left(Total\;N\;uptake\;in\;N/K\;fertilized\;plot\;uptake\right)}$$ (11)

$${RIUE}_{N/K}(kg\;{Mg}^{-1}grain\;yield)=\frac{{Uptake}_{\left(N/K\right)}}{Grain\;yield}$$ (12)

### 4.5. Development of artificial neural network (ANN) model for prediction of wheat yield

The ANNs competent of learning the data-set used during the training step, and then validate and train the network with parts of the initial data set that is used during the training step [105–107]. The ANNs are collection of a large number of inter-connected neurons, which are helpful device to forecast the concert of a simulation system, when the availability of experimental data-set is limited [105]. The ANNs are multi-layered feed forward completely connected network consists of an input layer, one or more hidden layers and an output layer [105, 108]. In the present study, we applied back propagation neural networks technique, and ANNs consisted of several layers of neurons which are inter-connected and then the weights were assigned to those inter-connections [106]. To simply clarify, weighted connections will permit to move among the layers wherein a node will accept data from the earlier layer and will compute the weighted sum for the net inputs (Eq 13).


$$t_{i}=\sum_{j=1}^{n}(w_{ij}x_{j}+b_{i})$$ (13)

Where, `n`= actual number of inputs, `w`= weight of the connection of the nodes that are `I`and `j`, `x`= input from `j`and `bi`= bias. The node outputs `oi`was computed from the transfer function `fi`using weighted values (Eq 14).


$$o_{i}=f_{i}(t_{i})$$ (14)

In back propagation neural network, input layer neurons distribute input ‘*X*_*i*_’ to the weights ‘$w_{ij}^{h}$’ of hidden layers without performing any computation. Outputs from hidden layer are computed in the first step and are passed by a following activation function (Eq 15).


$$Z_{j}=\partial_{j}(\sum_{i=1}^{P}W_{ij}^{h}+\gamma_{j}),j=1,2,3,den\;m$$ (15)

Where, ‘*Z*_*j*_’ = *activationfunction*, ‘∂_*j*_’= non-linear activation function used in a hidden layer and could be a hyperbolic tangent, sigmoid or logistic function. ‘*P’*= input number, ‘h’= symbol for hidden layer and ‘*γ*_*j*_’= j^th^ error term.

The ANN forecasting model is formulated as Eq 16.


$$X_{t+T+(m-1)\Gamma }^{F}=f(X_{t},w,\theta ,m,h)=\theta_{0}+\sum_{j=1}^{h}W_{j}^{out}\;\phi (\sum_{i=1}^{m}W_{ji}X_{t+(i-1)\Gamma +\theta_{j}})$$ (16)

Where, ‘*ϕ*’ is the transfer function, ‘*W*_*ji*_’ = weights describing connections between the ‘*i*^*th’*^node of the input layer and the ‘j^th^ ’node of the hidden layer, ‘*θ*_*j*_’ = biases related to the hidden layer, ‘$W_{j}^{out}$’ = weights related to connection between the ‘j^th^’node of the hidden layer and node of the output layer and ‘*θ*_0_’ = bias at the output layer. Therefore, to apply Eq 14 for wheat yield prediction, a suitable training algorithm was required to optimize values of ‘w’and ‘*θ*’. In the present study, ANNs provided with Levenberg–Marquardt training algorithm and hyperbolic tangent sigmoid transfer functions was used as a point of reference to examine model inputs in terms of root mean square error (RMSE), mean absolute error (MAE) and mean absolute percentage error (MAPE).

To simulate wheat grain yield (Mg ha^-1^) of the experimental data-set, ten different input layers (viz. grain N uptake, straw N uptake, grain K uptake, straw K uptake, total N uptake, total K uptake, SPAD value, green seeker value, RIUE_N_ and RIUE_K_) were used as input variables. The wheat grain yield was chosen as desired output parameter. The experimental data (pooled for two study years) were randomly divided into two sets viz. training data set (70%) and testing data set (30%).

### 4.6. Economic indices of wheat production

The mean cost of cash inputs (MCCIs) was estimated as sum of expenditure incurred for the purchase of inputs (US$ ha^-1^), e.g., seed, fertilizers, insecticides, fungicides, herbicides, etc. and labor cost for different field operations (Eq 17).


$$MCCIs(US\$\;ha^{-1})={\Sigma C}_{1,2,3,\ldots \ldots n}$$ (17)

Where C_1,2,3…._, represents cost for different inputs and labor.

The mean gross returns (MGRs) were estimated as a product of grain yield (Mg ha^-1^) under different treatments and minimum support price (MSP) of produce (rice, wheat) fixed by Government of India (US$ Mg^-1^) (Eq 18).


$$MGR(US\$\;ha^{-1})=Grain\;yield\;x\;MSP$$ (18)

Mean net returns (MNR) were estimated as the difference in MGR and MCCI (Eq 19).


$$\mathrm{MNRs}({\mathrm{US\$}\;\mathrm{ha}}^{-1})=\mathrm{MGRs}-\mathrm{MCCIs}$$ (19)

MCCIs, MGRs and MNRs were computed by converting Indian Rupee (INR) to United States Dollar (US$), considering 1US$ = 70 INR.

The benefit-cost (B-C) ratio was estimated as a ratio of MGRs and the MCCIs. The gross returns above the fertilizer cost (GRAFC) for wheat were estimated as the difference in between MGRs and amount (A) of N, P and K applied (kg ha^-1^) and price of N, P and K (US$ kg^-1^) as per treatment (Eq 20).


$$\mathrm{GRAFC}({\mathrm{US\$}\;\mathrm{ha}}^{-1})=[\mathrm{MGRs}]-[A_{\left(N+P+K\right)}\;{x\;\mathrm{price}}_{\left(N+P+K\right)}]$$ (20)

Where, ‘A_(N+P+K)_ ’represents amount of N+P+K applied and ‘price_(N+P+K)_’represents the market price of N+P+K. These estimations were based on market price of US$ 84.4 and 242.9Mg^-1^ for urea and MOP, respectively.

The economic efficiency was determined by dividing average net returns (ANR, US$ ha^-1^) from crop under different fertilizer treatments by crop duration (d) (Eq 21).


$$\mathrm{Economic}\;\mathrm{efficiency}\;({\mathrm{US\$}\;\mathrm{ha}}^{-1}d^{-1})=\frac{\mathrm{Mean}\;\mathrm{net}\;\mathrm{returns}\;(\mathrm{MNRs})}{\mathrm{Mean}\;\mathrm{crop}\;\mathrm{duration}}$$ (21)

The returns on investment (ROI) on fertilizers were estimated as a ratio of MGRs and total cost of fertilizers using Eq 22.


$$\mathrm{ROI}\;({\mathrm{US\$}\;\mathrm{ha}}^{-1})=\frac{\mathrm{MGRs}\;({\mathrm{US\$}\;\mathrm{ha}}^{-1})}{\mathrm{Total}\;\mathrm{cost}\;\mathrm{of}\;\mathrm{fertilizers}\;({\mathrm{US\$}\;\mathrm{kg}}^{-1})}$$ (22)

### 4.7. Statistical analysis

The data were analyzed using analysis of variance for the split plot design. All data-sets were analyzed using analysis of variance (ANOVA) and the differences between the means of treatment were separated by the least significant difference at the level of significance *p*<0.05 using IRRISTAT package [109]. The correlation matrix was developed in R software (R core team 2013). The step-wise multiple regression analysis was performed with SPSS 22.0 for Windows (IBM SPSS Inc., Chicago, U.S.A.). To develop ANN model for the prediction of wheat grain yield, MATLAB M-File environment version of MATLAB (R2017a, 9.2.0.538062) was used and program was written and run with Levenberg Marquardt algorithm. The statistical parameters viz. coefficient of determination (R^2^), RMSE, MAE and MAPE were calculated using following equations (Eqs 23–26). The correspondence between the measured and predicted root biomass of rice and wheat was graphically shown using 1:1 correspondence (X = Y).


$$R^{2}=1-(\frac{\sum (t_{i}-z_{i}{)}^{2}}{\sum t_{i}^{2}})$$ (23)

$$MAE=\frac{\sum \left|t_{1-}z_{1}\right|}{n}$$ (24)

$$RMSE=\sqrt{\frac{\sum (t_{i}-z_{i}{)}^{2}}{n}}$$ (25)

$$MAPE=\frac{1}{n}\sum |\frac{t_{i}-z_{i}}{t_{i}}|X\;100$$ (26)

Where, ‘n’= number of data points in the data set and ‘t’= actual output, ‘z’= predicted output. The significance of regression coefficients (slope and intercept) and coefficient of determination (R^2^) was tested using students’ T and F-test, respectively.

## 5. Conclusions

Higher N fertilizer application ensured higher crop yield and N accumulation, cause potential N losses and pollute source, but was not necessary to achieve optimal crop production. However, an increase in N supply did not affect the grain yield by increased K fertilization under sufficient available-K content in illitic soils. The higher rate of N and K fertilizer application decreased nutrient use efficiencies and fertilizer productivity. It is essential to increase NUE by reducing the input of N fertilizer and increasing the N absorption of crops, and to improve the sustainability of crop production. This study would help policy makers consider artificial neural network model and economic indices of wheat production suitable for up-scaling and large-scale adoption by smallholder farmers.
